The article "Risk Prediction of Maxillary Canine Impaction among 9-10-Year-Old Malaysian Children: A Radiographic Study" was published in 2022. Journal: Biomed Res Int.

# Risk Prediction of Maxillary Canine Impaction among 9-10-Year-Old Malaysian Children: A Radiographic Study

**DOI:** 10.1155/2022/5579243

**Published:** 2022-09-09

**Authors:** Ahmad Faisal Ismail, Nur Farhana Auni Sharuddin, Nur Hafizah Asha'ari, Mohd Adli Md Ali, Iswan Zuraidi Zainol, Lamis Hejab Alotaibi, Sreekanth Kumar Mallineni

**Affiliations:** ^1^Department of Paediatric Dentistry and Dental Public Health, Kulliyyah of Dentistry, International Islamic University Malaysia, Malaysia; ^2^Kulliyyah of Dentistry, International Islamic University Malaysia, Malaysia; ^3^Kulliyyah of Science, International Islamic University Malaysia, Malaysia; ^4^Department of Orthodontics, Kulliyyah of Dentistry, International Islamic University Malaysia, Malaysia; ^5^Department of Preventive Dental Science, College of Dentistry, Majmaah University, Al Majmaah 11952, Saudi Arabia; ^6^Center for Transdisciplinary Research (CFTR), Saveetha Institute of Medical and Technical Sciences, Saveetha Dental College, Saveetha University, Chennai, 600077 Tamil Nadu, India; ^7^Division for Globalization Initiative, Liaison Center for Innovative Dentistry Graduate School of Dentistry, Tohoku University, Sendai, Japan

## Abstract

**Background:**

Early diagnosis and interceptive treatment of the maxillary canine impaction is crucial as it reduces treatment complexity and decreases complications and adverse outcomes. *Aim and Objectives*. To determine the mean maxillary canine position among 9-10-year-old children and predict the risk of impaction of the maxillary canines. *Methodology*. Panoramic radiographs (PANs) of 289 healthy children aged between 9 and 10 years were observed where the average position of maxillary canines was related to the lateral incisor, sector locations, and angulations to the bicondylar line were traced. The average position was obtained by using descriptive statistics. One sample Wilcoxon signed-rank test is done to predict the risk of canine impaction by comparing the data obtained to the average position from prior studies.

**Results:**

A total of 289 PANs (126 males and 163 females) were utilized for the analysis. The findings showed that the average position of the maxillary canines in our population was statistically different from the average position of nonimpacted canines in previous studies. However, on average, more than 85% of canines in our population were still located within the safe range of satisfactory position, with females showing slight predominance outside of the acceptable range. The mean scores of the angles between the right canine and lateral incisor were significantly higher among females than males (*p* = 0.001). Similarly, females had a significantly higher mean angle of the left canine than males (*p* < 0.001). In regard to the angles between the bicondylar line and permanent maxillary canine, the mean scores were not significantly different (*p* > 0.05) on both the left and right side.

The article "Risk Prediction of Maxillary Canine Impaction among 9-10-Year-Old Malaysian Children: A Radiographic Study" was published in 2022. Journal: Biomed Res Int.

**Conclusion:**

There is a low risk of impaction of maxillary canines in the Malaysian population. However, more retrospective studies using more radiographic and clinical indicators need to be done to confirm the risk of impaction further.

## 1. Introduction

Maxillary canines are considered the cornerstone of the maxillary arch since they serve a pivotal role in the smile's aesthetic appearance and the occlusion's functional aspect. It may be because it is the tooth with the longest root and has good bony support [1]. Besides that, its long path of eruption and the lengthy development period causes it to be one of the last teeth to erupt. Though not as common as third molar impaction, the deleterious effects of late diagnosis of canine impaction make its early intervention an extremely crucial topic to be discussed [2]. Aside from creating aesthetic and functional problems, canine impaction can result in root resorption of neighboring teeth, necessitating surgical or orthodontic treatment for repositioning the impacted tooth to a favorable position. More complex displacements may pass unnoticed if not carefully evaluated and escape the time frame of early intervention [2, 3].

Mavreas and Athanasiou [4] reported that the analyzing factors responsible for the success of orthodontic treatment concluded that increased age and severity of impaction affect the complexity of treatment. Therefore, the most desirable approach for managing impacted canines is early diagnosis and the interception of potential impaction [5]. Palpation of the canine bulge in the buccal sulcus from 10 to 11 years is a well-established method for identifying canine impaction [6]. Nonetheless, various studies had been done to diagnose impacted canines early through panoramic radiographs and showed a notable degree of success [4–7]. Consequently, it has been reported that panoramic radiographs are a valuable tool for early prediction [7, 8]. The early observation of canine impaction through routine panoramic radiographs by general practitioners in Malaysia is not accustomed, considering the degree of seriousness of this disorder in the Malaysian community is not yet discussed. However, there are none of the studies reported on the investigation of maxillary canine position in the Malaysian population. Henceforth, the study is aimed at determining the mean maxillary canine position among 9-10 years old children and at predicting the risk of impaction of the maxillary canines.

The article "Risk Prediction of Maxillary Canine Impaction among 9-10-Year-Old Malaysian Children: A Radiographic Study" was published in 2022. Journal: Biomed Res Int.

## 2. Methodology

### 2.1. Study Design

This cross-sectional study was done according to a protocol that had been accepted and approved by the IIUM Human Research Ethics Committee (IREC) (ID no.: IREC 2021-006). All the data that were collected throughout this study will only be used for academic purposes. This study details would not be sold or reclaimed by other people without any permission, and all personal details of the child were protected to avoid misusage. This study was conducted at Polyclinic and Radiograph Unit (Kulliyyah of Dentistry, IIUM Kuantan). A convenience sampling method was used. The sample size was calculated using the following formula:

(1) $$\begin{array}{c} n=\frac{Z^{2}P\left(1-P\right)}{d^{2}}, \end{array}$$

where *n* is the sample size; *Z* value is the statistic for confidence level, 1.96 for 95% CI; *P* is the expected prevalence (estimated as 2%); *d* is the precision, where *d* = 0.02. The minimum sample size obtained was 188. Based on this value, a minimum of 188 panoramic radiographs (PANs) of children aged from 9 to 10 years, who attended Polyclinic Kulliyyah of Dentistry, Malaysia, were reviewed.

Children aged 9 to 10 years, who were fit and healthy and maxillary incisors, were fully erupted, with canines unerupted included in the study. Poor image quality and patients with pathology, such as syndromes, cleft lip, and palate, and severe abnormalities, and children with early extractions, orthodontic extrusion of the canine, or canines that are already erupted were excluded.

The average position of canines among children aged 9 to 10 years old was calculated as the average angulation between maxillary canines and the adjacent lateral incisors [9, 10] (3^2) (Figure 1). The position of unerupted maxillary canines and the adjacent lateral incisors, both left and right, was traced from 289 PANs. The angulations between the canines and the lateral incisors were then calculated using Python Programming. The average angulations were classified as either satisfactory or unsatisfactory based on the study by Almahdy et al. [11]. The average canine position is considered satisfactory if it is equal to or less than 30°. At more than 30°, the average canine position was classified as unsatisfactory. Next, the angulation and sector location of the canines were measured. The angular measurement was obtained in a manner; the most superior point of the condyle was selected as a landmark, and a bicondylar line was drawn as a horizontal reference line (Figure 2). The measurement was taken from the mesial angle formed between the constructed horizontal and the long axis of the unerupted canine, and the angles were then calculated using Python Programming. The position of the canine cusp tips was measured from the same tracing and classified into four sector locations as proposed by Lindauer et al. [12] as represented in Figure 3. Sector I represents the area distal to a line tangent to distal heights of the contour of the lateral incisor crown and root. Sector II is mesial sector I but distal to the bisector of the lateral incisor's long axis. Sector III is mesial to sector II but distal to mesial heights of the contour of lateral incisor crown and root. Sector IV includes all areas mesial to sector III. Prediction of the risk of canine impaction was made according to the results from a study by Warford et al. [13] and Quadras et al. [14] as shown below

Mean angulations:

Below 65°: unsatisfactory.

The article "Risk Prediction of Maxillary Canine Impaction among 9-10-Year-Old Malaysian Children: A Radiographic Study" was published in 2022. Journal: Biomed Res Int.

Equal and above 65°: satisfactory.

Sector locations:

Sector I: satisfactory.

Sector II, III, and IV: unsatisfactory.

From Figure 4, it can be demonstrated that the average position of canines in 9-10 years old children in the Malaysian population based on the 3 parameters (Figures 5 and 6) recorded in this study was located within a good position, where they are not located in close proximity or overlapping with the lateral incisors, nor they are in a position that shows a concerning path of eruption.

### 2.2. Data Analysis

All the available PANs were analyzed to determine the average position, angular measurements, and sector locations of the unerupted maxillary canines. Cohen's kappa was used for intraexaminer reliability. The average position was calculated as average angles between axes of the unerupted canines and the lateral incisors (3^2). Descriptive statistics were then applied to the angulations and sector locations to obtain the mean, standard deviation, median, and range. Mann–Whitney *U* test was used to analyze the significant differences between male and female patients for each parameter with the significance (*α*) value set at 0.05. Wilcoxon signed-rank test was used to detect the significant differences between the median of the study and the hypothetical mean of the previous study to predict the risk of impaction of those canines. SPSS (IBM SPSS Statistics for Windows, Version 20.0. Armonk, NY: IBM Corp) was used to analyze all the data.

## 3. Results

A total of 289 PANs (126 males and 163 females) were utilized for the analysis. Hence, 578 canines were analyzed cumulatively with an equal number of left and right canines of 289. Assessment for good intraexaminer reliability with Cohen's kappa analysis yielded a result of *κ* = 0.84.  Table 1 shows the descriptive statistics of the right and left maxillary canines. We can observe that both the mean and median of the angle between lateral incisor-canine and the angle between bicondylar line-canine are higher in the left canine compared to the right canine. Based on 3^2 angulation, higher mean and median were found in the female population compared to males. However, lower observed mean and median were found in the female population in terms of bicondylar angulation. The finding of our study indicates that the sector locations of unerupted canine cusp tips are primarily located in the sector I.

The article "Risk Prediction of Maxillary Canine Impaction among 9-10-Year-Old Malaysian Children: A Radiographic Study" was published in 2022. Journal: Biomed Res Int.

The frequency of the sector locations of the unerupted canine cusp tip in relation to the lateral incisor was summarized in Table 2. From the 289 PANs observed, the majority of both right and left canine cusp tips are located in sector I with a percentage of 90.7% and 86.5%, respectively, followed by sector II with a percentage of 7.3% on the right and 12.8% on its left. Besides that, a total of 5 teeth were observed in sector III and three teeth in sector IV; however, none of them was found on the left side in sector III.

The female predilection (20.91 ± 11.238) was found higher for right side Li-C angle than their male (16.83 ± 10.63) counterparts (*p* = 0.001) as described in Table 3. Females had a significantly higher mean angle of the left canine than males (*p* < 0.001). In regard to the angles between the bicondylar line and permanent maxillary canine, the mean scores were not significantly different (*p* > 0.05) on both left and right sides. However, the mean is still higher in males compared to females.

Our findings in Table 4 show that the average position of the maxillary canines in our population based on the parameters recorded, with the exception of the bicondylar right angle, is statistically different from the theoretical mean values of nonimpacted canines in previous studies, with *p* values less than 0.05. However, based on Table 5, on average, at least 70% of canines in our population are still located within the safe range of satisfactory position. Therefore, this finding might suggest that the canine position in our population is not a high-risk position for impaction. From another perspective, in each of the recorded parameters, females show a higher percentage of being located outside of the satisfactory position than males. Apart from that, left canines also show a slightly higher percentage compared to right canines within the unsatisfactory range. Out of all the parameters recorded, the bicondylar angle shows the least percentage of canines that is located within the satisfactory range, followed by the 3^2 angle and sector location.

## 4. Discussion

Maxillary canines are the most commonly impacted teeth, excluding the third molars. Numerous studies have been done on various populations globally to identify its incidences, such as in South China, Japan, and Italy [15–17]. The results cumulatively showed a range of 1-3% [18–21]. Even though it might seem like it affects a relatively small proportion of people, it is speculated that in individual orthodontic practice, the incidence may be higher [22]. This anomaly also shows a female predominance in various studies published in the literature with the condition affecting female patients 2.3 to 3 times more frequently than males [23–26]. Prior studies [24, 27–29] also found that left maxillary canines are more frequently affected compared to right canines. The present study may reflect the findings of these previous studies, where the females and left canines in this study are more predominant within the unsatisfactory range of position compared to males and right canines, respectively.

The article "Risk Prediction of Maxillary Canine Impaction among 9-10-Year-Old Malaysian Children: A Radiographic Study" was published in 2022. Journal: Biomed Res Int.

Despite various prevalence figures mentioned above, the etiology of impacted maxillary canines remains uncertain. A single or exclusive cause cannot fully determine the maxillary permanent canine impaction's outcome and could be multifactorial [30]. The contributing factors can be either general or local [25]. Examples of general factors are if the patient has systemic diseases such as endocrine deficiencies, any febrile diseases, and if the patient has a history of radiation exposure. On the other hand, the local contributing factors that cause canine impaction include the discrepancies between tooth size and the arch length, any retained deciduous canine or failure of resorption of the primary canine root, and early loss of the deciduous canine. Peck et al. [31] reported that missing or peg-shaped lateral incisors and abnormal position of the tooth bud play a role in determining the impaction of permanent maxillary canine. Other anomalies such as the presence of alveolar cleft, ankylosis of the permanent canine, cystic or neoplastic formation, and dilacerations of the root also may cause disturbances to the eruption path, thus causing impaction of those canines. Along with it, evidence of genetic predisposition and familial occurrence of impacted canines were also found [32].

Prior studies [8–10, 17, 18, 20] investigated on impacted canines and reported that palatally displaced canines (PDC) and buccally displaced canines (BDC) have different etiopathogenesis. BDC is thought to be a result of crowding [29] and PDC, however, often occurs in patients with sufficient space in the maxillary arch for canine eruption [33]. The “guidance theory” refers to the lack of guidance by the adjacent teeth during the canine eruption, such as missing maxillary lateral incisors [34, 35]. The “genetic theory” explains that PDC is only one aspect of a general dental disorder that is genetic in origin and hereditary, which also causes other dental anomalies such as peg-shaped lateral incisors, cleft lip, and palate, and displaced premolars [17, 23, 24, 36–42]. In the present study, further analysis of the sample background and follow-up of the outcome of the canine position is either impacted buccally or palatally or not.

The article "Risk Prediction of Maxillary Canine Impaction among 9-10-Year-Old Malaysian Children: A Radiographic Study" was published in 2022. Journal: Biomed Res Int.

During patient history taking and examination, the dentist should suspect a potentially palatal impaction of permanent maxillary canine if the canine is not palpable in the buccal sulcus by the age of 10 to 11 years, and asymmetrical eruption pattern of canine is noted [6]. The early detection of signs of ectopic eruption of the canines will prevent impaction and its potential sequelae. Ericson and Kurol [43] also suggested that an early diagnosis and treatment of the palatally ectopic canine is essential for a successful outcome. Based on the algorithm for management of the ectopic canine, radiographic investigations are indicated in patients ten years old and above with no canine bulge seen or palpable to detect any pathology or if there is a missing permanent tooth bud. Otherwise, if there is evidence of the canine presence and favorable for normal eruption, the child patient aged 10 to 13 years old might need an interceptive treatment and monitor their canine eruption for 12 months. Suppose, no permanent successor is present in the radiographic assessment. In that case, it is a sign that the patient might need a referral for specialist consultation and management and subsequent definitive orthodontic treatment if required. If not intercepted early, the impacted canine will cause several possible complications, such as root resorption of the adjacent teeth, formation of a dentigerous cyst, infection, and referred pain [26, 44–46]. Ravi et al. [47] reported that the sector classification, the angle formed by the long axis of the canine and the midline, an angle formed by the long axis of the canine and the lateral incisor, and the perpendicular distance between the canine cusp tip to the occlusal plane and to the midline and an angle formed by the long axis of the canine and the occlusal plane are commonly used predictors for maxillary impaction. The authors also reported that PANs are the best tools for the prediction of maxillary canine impaction. In the present study, PANs for the prediction of canine impaction are in the maxillary arch. Dadgar et al. [48] reported that the head and neck skeletal anomalies or variants could be used for the prediction of palatal canines. The present study was not explicitly focused on palatal canines, and PANs were used for the analysis.

The article "Risk Prediction of Maxillary Canine Impaction among 9-10-Year-Old Malaysian Children: A Radiographic Study" was published in 2022. Journal: Biomed Res Int.

The findings in the present study showed that the average position of unerupted canines in the Malaysian population is statistically different from the theoretical average value of unerupted nonimpacted canines from previous studies. This suggests that the average unerupted canine position in the Malaysian population is unsatisfactory. However, this is probably because the theoretical mean values that are used to compare with the means obtained in this study consist of the mean values of unerupted nonimpacted canines' position from a sample of a different population from the present article. The present study consists of the Southeast Asian population, while the previous studies used in this comparison consist of the United States and South Asian populations. More retrospective studies using more radiographic and clinical indicators in the Southeast Asian population need to be done to confirm the risk of impaction. Other than that, in the present study, all outliers are included within the data analysis, to prevent the exclusion of children that are actually at high risk for impaction. This may also bring about the difference of average in the present study to the theoretical value. Therefore, the percentage of canines within the satisfactory or unsatisfactory range provides more significance in determining whether the position of unerupted canines in the Malaysian population is within a satisfactory and low-risk position. The study sample size is very small, and the findings were confined only to the Malaysian population. The study sample was hospital-based. Nonetheless, a follow-up of the subsequent canine position from the sample population should be conducted to confirm whether the unsatisfactory range in this study foreshadows canine impaction. These are considered potential limitations of the present study. Various treatments might be suggested for an individual on a case-by-case basis.

## 5. Conclusion

The majority of the maxillary permanent canine buds of Malaysian children of 9 to 10 years of age are in an acceptable position. An early prediction of maxillary canine is beneficial for the dentist to develop an appropriate treatment plan to avoid potential complications.

- On average, more than 85% of canines in our population were still located within the safe range of satisfactory position, with females showing slight predominance outside of the acceptable range
- The mean scores of the angles between the right canine and lateral incisor were significantly higher among females than males (*p* = 0.001), and females had a significantly higher mean angle of the left canine than males (*p* < 0.001)

The article "Risk Prediction of Maxillary Canine Impaction among 9-10-Year-Old Malaysian Children: A Radiographic Study" was published in 2022. Journal: Biomed Res Int.

## Figures and Tables

**Figure 1:** Parameter 1 (angle A): the angle between the axis of the unerupted canine and the lateral incisor (3^2).

**Figure 2:** Parameter 2 (angle B): the angle between the bicondylar line and canine.

**Figure 3:** Parameter 3: the sector location of the canine—position of canine cusp tip in relation to the lateral incisors.

**Figure 4:** Average position of permanent canines among 9-10 years old children.

**Figure 5:** Showing parameters 1 and 2 traced on a panoramic radiograph.

**Figure 6:** Showing parameter 3 traced on panoramic radiograph.

**Table 1:** Descriptive details of right and left maxillary canines.

Parameter		3^2	Bicondylar	Sector
Right	Mean (SD)	19.204 (11.197) Male: 16.832 (10.637) Female: 20.919 (11.238)	69.654 (11.346) Male: 70.604 (10.612) Female: 68.919 (11.863)	
	Median (range)	17.598 (84.469) Male: 15.587 (84.469) Female: 19.358 (68.38)	70.391 (156.572) Male: 71.397 (72.905) Female: 69.385 (76.425)	1 (0)

Left	Mean (SD)	19.872 (9.991) Male: 17.622 (9.991) Female: 21.518 (9.624)	70.639 (10.671) Male: 71.640 (10.496) Female: 69.864 (10.773)	
	Median (range)	19.106 (74.916) Male: 17.095 (74.413) Female: 20.363 (55.810)	71.397 (161.899) Male: 72.402 (81.453) Female: 70.391 (67.745)	1 (0)

SD: standard deviation.

**Table 2:** Frequency data of sector location.

Sector	*n* (%)	
	Right	Left
I	262 (90.7%)	250 (86.5%)
II	21 (7.3%)	37 (12.8%)
III	5 (1.7%)	0
IV	1 (0.3%)	2 (0.7%)
Total	289	289

**Table 3:** Differences of radiographic parameters between males and females.

Parameters	*N*	3^2		Bicondylar	
		Mean (SD)	*p* values	Mean (SD)	*p* values
Right					
Male	126	16.832 (10.637)	0.001^∗^	70.604 (10.612)	0.147
Female	163	20.919 (11.238)		68.919 (11.863)	

Left					
Male	126	17.622 (9.991)	0.000^∗^	71.640 (10.496)	0.094
Female	163	21.518 (9.624)		69.864 (10.773)	

^∗^ *p* < 0.05; Mann–Whitney *U* test for two group comparison; SD: standard deviation.

**Table 4:** Differences of radiographic parameters between hypothetical mean and observed median values.

Parameters	*p* value
3^2 right	<0.001^∗^
3^2 left	<0.001^∗^
Bicondylar right	0.230
Bicondylar left	0.012^∗^

^∗^ *p* < 0.05; Wilcoxon signed-rank test for two studies comparison.

**Table 5:** Prediction of the risk of canine impaction.

Parameter		Angle, *n* (%)	Gender, *n* (%)	Mean (SD)	Median (range)
3^2	Right	≤30: 249 (86.2%)	M: 117 (92.9%) F: 132 (81.0%)	15.900 (6.842)	16.089 (29.665)
		>30: 40 (13.8%)	M: 9 (7.1%) F: 31 (19.0%)	39.771 (11.160)	35.698 (54.302)
	Left	≤30: 248 (85.8%)	M: 117 (92.9%) F: 131 (80.4%)	17.101 (7.153)	17.095 (29.162)
		>30: 41 (14.2%)	M: 9 (7.1%) F: 32 (19.6%)	36.630 (8.205)	34.190 (45.251)

Bicondylar	Right	<65: 85 (29.4%)	M: 29 (23%) F: 56 (34.4%)	56.676 (10.267)	59.832 (47.765)
		≥65: 204 (70.6%)	M: 97 (77%) F: 107 (65.6%)	75.061 (6.254)	74.916 (28.156)
	Left	<65: 71 (24.6%)	M: 21 (16.7%) F: 50 (30.7%)	56.987 (9.081)	60.335 (49.777)
		≥65: 218 (75.4%)	M: 105 (83.3%) F: 113 (69.3%)	75.085 (6.611)	74.413 (32.682)

Sector	Right	I: 262 (90.7%)	M: 116 (92.1%) F: 146 (89.6%)		1 (0)
		II, III, IV: 27 (9.3%)	M: 10 (7.9%) F: 12 (10.4%)		2 (2)
	Left	I: 250 (86.5%)	M: 114 (90.5%) F: 136 (83.4%)		1 (0)
		II, III, IV: 39 (13.5%)	M: 12 (9.5%) F: 27 (16.6%)		2 (2)

*n* = 289; SD: standard deviation.

The article "Risk Prediction of Maxillary Canine Impaction among 9-10-Year-Old Malaysian Children: A Radiographic Study" was published in 2022. Journal: Biomed Res Int.

## Data Availability

The raw data supporting the conclusions of this article will be made available by the authors without undue reservation.

## References

[1] Oral Health Division MOH Malaysia (2016). *Clinical Practice Guidelines: Management of the Palatally Ectopic Canine*.

[2] Motamedi M. H. K., Talesh K. T. (2005). Management of extensive dentigerous cysts. *British Dental Journal*.

[3] Alqerban A., Jacobs R., Lambrechts P., Loozen G., Willems G. (2009). Root resorption of the maxillary lateral incisor caused by impacted canine: a literature review. *Clinical Oral Investigations*.

[4] Mavreas D., Athanasiou A. E. (2008). Factors affecting the duration of orthodontic treatment: a systematic review. *European Journal of Orthodontics*.

[5] Bedoya M. M., Park J. H. (2009). A review of the diagnosis and management of impacted maxillary canines. *The Journal of the American Dental Association*.

[6] Ericson S., Kurol J. (1986). Longitudinal study and analysis of clinical supervision of maxillary canine eruption. *Community Dentistry and Oral Epidemiology*.

[7] Margot R., Maria C. D., Ali A., Annouschka L., Anna V., Guy W. (2020). Prediction of maxillary canine impaction based on panoramic radiographs. *Clinical and Experimental Dental Research*.

[8] Mehta F., Jain M., Verma S. (2022). Morphological comparison of the maxillary arch in buccal and palatal canine impaction among Asian population of Gujarati origin: a hospital-based study. *Healthcare*.

[9] Alqerban A., Storms A. S., Voet M., Fieuws S., Willems G. (2016). Early prediction of maxillary canine impaction. *Dentomaxillofacial Radiology*.

[10] Sajnani A. K., King N. M. (2012). Early prediction of maxillary canine impaction from panoramic radiographs. *American Journal of Orthodontics and Dentofacial Orthopedics*.

[11] Almahdy A., Alqerban A., Aljasir O., Alsaghir Z., Alhammad S. (2018). Early radiographic features of maxillary canine impaction for orthodontically diagnosed children aged between 8-14 years old. *Journal of Clinical and Diagnostic Research*.

The article "Risk Prediction of Maxillary Canine Impaction among 9-10-Year-Old Malaysian Children: A Radiographic Study" was published in 2022. Journal: Biomed Res Int.

[12] Lindauer S. J., Rubenstein L. K., Hang W. M., Andersen W. C., Isaacson R. J. (1992). Canine impaction identified early with panoramic radiographs. *The Journal of the American Dental Association*.

[13] Warford J. H., Grandhi R. K., Tira D. E. (2003). Prediction of maxillary canine impaction using sectors and angular measurement. *American Journal of Orthodontics and Dentofacial Orthopedics*.

[14] Quadras D. D., Krishna Nayak U. S., Ravi M. S., Pujari P. (2017). Early prediction of maxillary canine impaction using sectors and angular measurement-a radiographic study. *Manipal Journal of Dental Sciences*.

[15] Sajnani A. K., King N. M. (2014). Prevalence and characteristics of impacted maxillary canines in southern Chinese children and adolescents. *Journal of Investigative and Clinical Dentistry*.

[16] Takahama Y., Aiyama Y. (1982). Maxillary canine impaction as a possible microform of cleft lip and palate. *European Journal of Orthodontics*.

[17] Sacerdoti R., Baccetti T. (2004). Dentoskeletal features associated with unilateral or bilateral palatal displacement of maxillary canines. *Angle Orthodontics*.

[18] Bishara S. E. (1998). Clinical management of impactedmaxillary canines. *Seminars in Orthodontics*.

[19] Ericson S., Kurol J. (1987). Radiographic examination of ectopically erupting maxillary canines. *American Journal of Orthodontics and Dentofacial Orthopedics*.

[20] Kramer R. M., Williams A. C. (1970). The incidence of impacted teeth. *Oral Surgery Oral Medicine Oral Pathology*.

[21] Thilander B., Myrberg N. (1973). The prevalence of malocclusion in Swedish schoolchildren. *European Journal of Oral Sciences*.

[22] Ferguson J. W. (1990). Management of the unerupted maxillary canine. *British Dental Journal*.

[23] Becker A., Chaushu S. (2015). Etiology of maxillary canine impaction: a review. *American Journal of Orthodontics and Dentofacial Orthopedics*.

[24] Mercuri E., Cassetta M., Cavallini C., Vicari D., Leonardi R., Barbato E. (2013). Dental anomalies and clinical features in patients with maxillary canine impaction. *The Angle Orthodontist*.

[25] Cooke J., Wang H. L. (2006). Canine impactions: incidence and management. *The International Journal of Periodontics & Restorative Dentistry*.

[26] Bishara S. E., Ortho D. (1992). Impacted maxillary canines: a review. *Am J Orthod Dentofacial Orthopaedics*.

[27] Syrynska M., Budzynska A. (2008). The incidence of uni- and bilateral impacted maxillary canines and their position in dental arch depending on gender and age. *Annales Academiae Medicae Stetinensis*.

[28] Peck S., Peck L., Kataja M. (1994). The palatally displaced canine as a dental anomaly of genetic origin. *The Angle Orthodontist*.

The article "Risk Prediction of Maxillary Canine Impaction among 9-10-Year-Old Malaysian Children: A Radiographic Study" was published in 2022. Journal: Biomed Res Int.

[29] Jacoby H. (1983). The etiology of maxillary canine impactions. *American Journal of Orthodontics*.

[30] Alqerban A., Jacobs R., Fieuws S., Willems G. (2015). Radiographic predictors for maxillary canine impaction. *American Journal of Orthodontics and Dentofacial Orthopedics*.

[31] Peck S., Peck L., Kataja M. (1996). Prevalence of tooth agenesis and peg-shaped maxillary lateral incisor associated with palatally displaced canine (PDC) anomaly. *American Journal of Orthodontics and Dentofacial Orthopedics*.

[32] Camilleri S., Lewis C. M., McDonald F. (2008). Ectopic maxillary canines: segregation analysis and a twin study. *Journal of Dental Research*.

[33] Barbato E., Proietti D., Malagola C. (1990). Evaluation of upper arch dimensions in subjects with palatally impacted canines. *Mondo Ortodontico*.

[34] Al-Nimri K. S., Bsoul E. (2011). Maxillary palatal canine impaction displacement in subjects with congenitally missing maxillary lateral incisors. *American Journal of Orthodontics and Dentofacial Orthopedics*.

[35] Becker A., Sharabi S., Chaushu S. (2002). Maxillary tooth size variation in dentitions with palatal canine displacement. *The European Journal of Orthodontics*.

[36] Mallineni S. K., Jayaraman J. (2021). A novel report of dental development pattern in a 3-year-old girl with three congenitally missing primary canines: a review of the literature and a case study. *Journal of the Indian Society of Pedodontics and Preventive Dentistry*.

[37] Baccetti T., Leonardi M., Giuntini V. (2010). Distally displaced premolars: a dental anomaly associated with palatally displaced canines. *American Journal of Orthodontics and Dentofacial Orthopedics*.

[38] Becktor K. B., Steiniche K., Kjaer I. (2005). Association between ectopic eruption of maxillary canines and first molars. *European Journal of Orthodontics*.

[39] Camilleri S. (2005). Maxillary canine anomalies and tooth agenesis. *European Journal of Orthodontics*.

[40] Leonardi R., Peck S., Caltabiano M., Barbato E. (2003). Palatally displaced canine anomaly in monozygotic twins. *Angle Orthodontics*.

[41] Leifert S., Jonas I. E. (2003). Dental anomalies as a microsymptom of palatal canine displacement. *Journal of Orofacial Orthopedics*.

[42] Nirmala S., Mallineni S. K., Nuvvula S. (2013). Pre-maxillary hypo-hyperdontia: report of a rare case. *Romanian Journal of Morphology and Embryology*.

[43] Ericson S., Kurol J. (1988). Early treatment of palatally erupting maxillary canines by extraction of the primary canines. *The European Journal of Orthodontics*.

[44] Ericson S., Kurol J. (1988). Resorption of maxillary lateral incisors caused by ectopic eruption of the canines. A clinical and radiographic analysis of predisposing factors. *American Journal of Orthodontics and Dentofacial Orthopedics*.

The article "Risk Prediction of Maxillary Canine Impaction among 9-10-Year-Old Malaysian Children: A Radiographic Study" was published in 2022. Journal: Biomed Res Int.

[45] Rimes R. J., Mitchell C. N. T., Willmot D. R. (1997). Maxillary incisor root resorption in relation to the ectopic canine: a review of 26 patients. *European Journal of Orthodontics*.

[46] Laurenziello M., Montaruli G., Gallo C. (2017). Determinants of maxillary canine impaction: retrospective clinical and radiographic study. *Journal of Clinical and Experimental Dentistry*.

[47] Ravi I., Srinivasan B., Kailasam V. (2021). Radiographic predictors of maxillary canine impaction in mixed and early permanent dentition–a systematic review and meta-analysis. *International Orthodontics*.

[48] Dadgar S., Alimohamadi M., Rajabi N., Rakhshan V., Sobouti F. (2021). Associations among palatal impaction of canine, sella turcica bridging, and ponticulus posticus (atlas arcuate foramen). *Surgical and Radiologic Anatomy*.

